This article has been retracted.

# Exosomal long non-coding RNA UCA1 functions as growth inhibitor in esophageal cancer

**DOI:** 10.18632/aging.103911

**Published:** 2020-10-29

**Authors:** Zijiang Zhu, Huilin Wang, Yao Pang, Hongxia Hu, Hongyi Zhang, Wenhao Wang

**Affiliations:** 1 Department of Thoracic Surgery, Gansu Provincial Hospital, Lanzhou, Gansu, China

**Keywords:** esophageal cancer, exosome, lncRNA UCA1, progression, biomarker

## Abstract

Purpose: Esophageal cancer is a highly lethal and broad-spreading malignant tumor worldwide. Exosome-carrying lncRNAs play an essential role in the pathogenesis of various cancers.

Results: The results revealed that the expression of UCA1 was decreased in esophageal cancer tissues and plasma exosomes. UCA1 was enriched in exosomes, and exosomal UCA1 was a promising biomarker for the diagnosis of esophageal cancer with 86.7% sensitivity and 70.2% specificity. Overexpression of UCA1 played anticancer roles in esophageal cancer cells through inhibiting cell proliferation, invasion and migration, and colony formation. Also, exosomal UCA1 was taken up by esophageal cancer cells and inhibited the progression of esophageal cancer *in vitro* and tumor growth *in vivo*. Furthermore, exosomal UCA1 could directly target miRNA-613 in esophageal cancer cells.

Conclusions: The results suggested that exosomal UCA1 inhibits tumorigenesis and progression of esophageal cancer *in vitro* and *in vivo*, and might be a promising biomarker for esophageal cancer.

Patient and Methods: In this study, we determined the expression of UCA1 in esophageal cancer tissues, plasma exosomes of patients with esophageal cancer. We determined the potential of exosomal UCA1 as a biomarker and its effect on the pathogenesis and progression of esophageal cancer *in vitro* and *in vivo*.

## INTRODUCTION

Esophageal cancer is one of the most wide-spreading malignant tumors of the digestive tract all over the world, with 14% 5-years survival rate [1, 2]. As one of the high-incidence countries of esophageal cancer, it is estimated that approximately 291,238 esophageal cancer-related deaths were reported in China in 2011 [3]. To date, several available treatments, such as surgical treatment, radiation therapy, chemotherapy, as well as the combined treatment, have improved the survival rate of esophageal cancer [4, 5]. However, there was little improvement in mortality over the past few decades. The majority of patients with esophageal cancer are not suitable for surgical treatment because many cases are undiagnosed until the disease develops to the advanced stage. Also, recurrence, radio- and chemo-resistance, and the metastatic property result in the poor prognosis of esophageal cancer [6]. Currently, a lack of a clear understanding of mechanisms underlying the pathogenesis and progression are primary obstacles in developing effective diagnostic and therapeutic options for esophageal cancer.

Long non-coding RNAs (lncRNAs) are a set of non-coding RNAs with greater than 200 nucleotides in length [7]. Accumulating evidence suggests that lncRNAs play an essential role in a wide variety of biological processes, such as cell cycle, transcription, translation, methylation, and apoptosis [8]. Also, considerable attention from researchers worldwide has been paid to the function of lncRNAs in cancer pathogenesis, including gastric cancer [9], cervical cancer [10], glioblastoma multiforme [11], and esophageal cancer [12]. In the past decade, growing studies have reported that exosomes are a class of lipid bilayer-enclosed extracellular vesicles with a size range of 40-150 nm [13]. Exosomes can be released by all cell types and play a significant role in cell-to-cell communication by transporting bioactive molecules, including proteins, metabolites, DNAs, and RNAs [14, 15]. Therefore, it has been well documented that exosome-mediated intercellular communication not only participates in the regulation of normal physiological processes, but also in various pathological processes of many diseases, including cancers [13, 16], neurodegenerative diseases [17], and cardiovascular disease [18]. Furthermore, due to the stability and broad presence of exosomes in various bodily fluids, exosome-carrying cargos have a promising potential to serve as a biomarker for early diagnosis of various diseases [19, 20].

In this study, we screened the expressions of twenty lncRNAs that have been reported to be associated with multiple cancers in esophageal cancer tissues and plasma exosomes. Of which, our observations demonstrated that lncRNA UCA1 was downregulated in both esophageal tissues and exosomes from the plasma of patients with esophageal cancer. As one of the well-studied lncRNAs in cancer, UCA1 has been reported to exert an essential role in cell proliferation, tumor growth, invasion, and epithelial-mesenchymal transition in esophageal cancer [21–23]. However, the function of exosomal UCA1 in esophageal cancer remains unclear. Thus, this study aimed to investigate the effect of exosomal UCA1 in the pathogenesis of esophageal cancer and if exosomal UCA1 can be applied as a diagnostic biomarker for esophageal cancer.

## RESULTS

### Patient characteristics and expression of UCA1 in esophageal cancer tissues

In this study, we collected information about thirty esophageal cancer cases as well as thirty healthy controls, and their characteristics were summarized in Table 1. Of which, we found that there were differences between cancer cases and healthy controls in pack-years of smoking (p= 0.045) and smoking status (p= 0.031). In addition, the majority of cancer cases were in clinical grade 0-II (76.6%) and with lymph nodes (66.7%). Then, twenty tumor-associated lncRNAs were selected based on previous studies [22, 24, 25], and their expressions were determined in esophageal cancer tissues. The results revealed that the levels of GAS5, H19, and MEG3 were increased, while UCA1 was decreased in esophageal cancer tissues relative to those of adjacent healthy tissues (Figure 1A, 1B).

**Table 1:** Characteristics of patients with esophageal cancer.

**Characteristics**	**Control (n = 30) N (%)**	**Case (n = 30) N (%)**	***P***
**Age (mean ± SD)**	63.1 ± 6.8	64.3 ± 7.2	0.504
**Sex**			
**Male**	21 (70.0)	17 (56.7)	
**Female**	9 (30.0)	13 (43.3)	
**Pack-year (mean ± SD)**	47.4 ± 6.9	28.1 ± 5.8	0.045
**Smoking**			0.031
**Never**	14 (46.7)	6 (20.0)	
**Ever**	16 (53.3)	24 (80.0)	
**Drink alcohol**			0.321
**Yes**	13 (43.3)	14 (46.7)	
**No**	17 (56.7)	16 (53.3)	
**Nodal status**		
**Yes**		20 (66.7)	
**No**		10 (33.3)	
**Cancer stage**		
**0-II**		23 (76.7)	
**III-IV**		7 (23.3)	
**Histology**		
**Adenocarcinoma**		19 (63.0)	
**Squamous cell carcinoma**		9 (30.0)	
**Adenosquamous carcinoma**		2 (7.0)	

Student’s t-test for age between controls and cases.

Two-sided χ2 for other characteristics between controls and cases.

**Figure 1:** **Expression of UCA1 in esophageal cancer tissues.** (**A**, **B**) Expressions of candidate lncRNAs in esophageal cancer tissues (Tumor) and paired normal tissues (Control) (n=15). (**C**) Morphology and size of exosomes derived from the plasma of patients with esophageal cancer (Tumor) or control subjects (Control). Scale bar = 200 nm. (**D**) Protein expressions of exosomal markers TSG101 and CD63 in exosomes derived from the plasma of patients with esophageal cancer (Tumor) or control subjects (Control). (*) denotes the difference between groups (*P*<0.05). Each experiment had a minimum of three replicates per treatment group.

### Expression of UCA1 in plasma exosomes isolated from patients with esophageal cancer

Plasma exosomes derived from patients with esophageal cancer and healthy controls were isolated through ultracentrifugation-based assay. The characteristics of exosomes were determined by TEM and NTA assays. The results suggested that exosomes displayed a round shape, and the majority of exosomes were 120-150 nm in diameter (Figure 1C). Then, we performed western blots assay to detect the exosomal markers TSG101 and CD63, and the results revealed that both TSG101 and CD63 were highly enriched in exosomes derived from patients with esophageal cancer and healthy controls (Figure1D). Based on the observations in cancer tissues, we determined the expressions of GAS5, H19, MEG3, and UCA1 in plasma exosomes. The results showed that the exosomal UCA1 was significantly decreased in the exosomes from the plasma of esophageal cancer patients compared with those of healthy controls (Figure 2A). Furthermore, we performed ROC curves analysis to determine the potential of exosomal UCA1 as a non-invasive biomarker in esophageal cancer. As shown in Figure 2B, the AUC was 0.8522 (95% CI = 0.7559-0.9485) for exosomal UCA1. The sensitivity and specificity of exosomal UCA1 as a biomarker to predict the presence of esophageal cancer were 86.7% and 70.2%, respectively. It has been demonstrated that exosome-carrying cargos are stable under different conditions [26, 27]. Thus, we tested the stability of exosomal UCA1 in the plasma samples placed at room temperature for different times or experienced different freezing-thawing cycles. In both scenarios, the level of exosomal UCA1 did not alter in the different conditions (Figure 2C, 2D), indicating that exosomal UCA1 might be a potential biomarker for esophageal cancer.

**Figure 2:** **Expression of exosomal UCA1 in patients with esophageal cancer.** (**A**) Expression of exosomal UCA1 from the plasma of patients with esophageal cancer (Tumor) or control subjects (Control). (**B**) ROC curves analysis of exosomal UCA1. (**C**) Expression of exosomal UCA1 in the plasma samples placed at room temperature for 0 h, 4 h, 8 h, and 24 h, respectively. (**D**) Expression of exosomal UCA1 in the plasma samples after 0, 2, 3, 4 freezing-thawing cycles. (*) denotes the difference between groups (*P*<0.05). Each experiment had a minimum of three replicates per treatment group.

### Effect of overexpression of UCA1 on esophageal cancer cells

Given the findings that UCA1 was downregulated in both esophageal cancer tissues and plasma exosomes, we next aimed to investigate the effect of UCA1 on esophageal cancer cell lines EC18 and Kyse140. After transfecting with UCA1-expressing plasmids (vector-UCA1) or negative control plasmids (vector-NC), the levels of UCA1 were significantly upregulated in both esophageal cancer cell lines (Figure 3A). In the functional experiments, we found that the overexpression of UCA1 exerted an inhibitory role in cell proliferation in EC18 and Kyse140 cells (Figure 3B, 3C). Meanwhile, the invasive and migratory abilities were also suppressed by forced expression of UCA1 in esophageal cancer cells (Figure 3D, 3E). Additionally, EC18 and Kyse140 cells with overexpression of UCA1 showed a lower rate of colony formation (Figure 3F). Together, the results suggest that UCA1 is an antitumor factor for esophageal cancer.

**Figure 3:** **Effect of overexpression of UCA1 on esophageal cancer cells.** (**A**) Expression of UCA1 in esophageal cancer cell lines EC18 and Kyse140 transfected with UCA1-expressing plasmids (vector-UCA1) or negative control plasmids (vector-NC). (**B**, **C**) Cell viability of EC18 and Kyse140 cells transfected with UCA1-expressing plasmids (vector-UCA1) or negative control plasmids (vector-NC). Scale bar = 50 nm. (**D**) Invasive ability of EC18 and Kyse140 cells transfected with UCA1-expressing plasmids (vector-UCA1) or negative control plasmids (vector-NC). Scale bar = 50 nm. (**E**) Migratory ability of EC18 and Kyse140 cells transfected with UCA1-expressing plasmids (vector-UCA1) or negative control plasmids (vector-NC). Scale bar = 50 nm. (**F**) Colony formation ability of EC18 and Kyse140 cells transfected with UCA1-expressing plasmids (vector-UCA1) or negative control plasmids (vector-NC). (*) denotes the difference between groups (*P*<0.05). Each experiment had a minimum of three replicates per treatment group.

### Exosomal UCA1 participated in intercellular communication

To further investigate the role of UCA1, we then determined the distribution pattern of extracellular UCA1. In the cell culture mediums, the addition of RNaseA did not affect the level of UCA1, while the combination of RNaseA and Triton X-100 inhibited the level of UCA1 (Figure 4A). Thus, these observations implied that UCA1 was highly enriched in the membrane-surrounding environment. Then, we isolated exosomes from NEEC, EC18, and Kyse140 cell mediums, respectively. As mentioned above, the characteristics of exosomes were also verified by TEM and NTA assays (Figure 4B), as well as western blots assay (Figure 4C). Next, we determined the expression of UCA1 in both exosomes and exosome-releasing cells, and we found that the levels of UCA1 were higher in exosomes relative to the donor cells (Figure 4D). In addition, we observed that the levels of UCA1 were higher in NEEC-derived exosomes, compared to those derived from EC18, and Kyse140 cells (Figure 4E), which is consistent with our observations that UCA1 was increased in control healthy tissues (Figure 1A). Furthermore, by fluorescence staining assay, we found that NEEC-derived exosomes labeled fluorescent green were internalized by EC18 and Kyse140 cells whose nuclei were labeled fluorescent blue (Figure 4F). Also, the green-labeled exosomes were found to be highly enriched in the cytoplasm.

**Figure 4:** **Exosomal UCA1 participated in intercellular communication.** (**A**) Expression of UCA1 in the medium of NEEC, EC18, and Kyse140 cells treated with RNase (2 ug/ml) or the combination of RNase (2 ug/ml) and Triton X-100 (0.1%). (**B**) Morphology and size of exosomes derived from the medium of NEEC, EC18, and Kyse140 cells, respectively. Scale bar = 100 nm. (**C**) Protein expressions of exosomal markers TSG101 and CD63 in exosomes derived from the medium of NEEC, EC18, and Kyse140 cells, respectively. (**D**) Relative expressions of UCA1 in exosomes and exosome-releasing cells. (**E**) Relative expressions of UCA1 in exosomes derived from NEEC, EC18, and Kyse140 cells. (**F**) Exosomes derived from NEEC cells were taken up by EC18, and Kyse140 cells. Exosomes were labeled with PKH67 (green), and the nuclei were labeled with DAPI (blue). Scale bar = 25 nm. (*) denotes the difference between groups (*P*<0.05). Each experiment had a minimum of three replicates per treatment group.

### Effect of exosomal UCA1 on esophageal cancer cells

As found above, UCA1 could be shuttled from NEEC cells to EC18, and Kyse140 cells through exosome-mediated intercellular communication, we then attempted to investigate the effect of exosomal UCA1 on esophageal cancer cells. Firstly, we isolated exosomes from NEEC cells transfected with UCA1-expressing plasmids (UCA1-Exo) or negative control plasmids (control-Exo). Then, we cocultured EC18 and Kyse140 cells with UCA1-Exo or control-Exo and determined the expression of UCA1. The results showed that the levels of UCA1 were higher in EC18 and Kyse140 cells treated with UCA1-Exo, compared with those in cells treated with control-Exo (Figure 5A). Similar to the results showed in Figure 3, EC18, and Kyse140 cells treated with UCA1-Exo exhibited inhibited cell proliferation (Figure 5B, 5C), invasion (Figure 5D), migration (Figure 5E), and colony formation (Figure 5F), compared with those treated with control-Exo. Collectively, exosomal UCA1 plays a significant anticancer role in esophageal cancer *in vitro*.

**Figure 5:** **Effect of exosomal UCA1 on esophageal cancer cells.** (**A**) Expression of UCA1 in EC18 and Kyse140 cells treated with exosomes derived from NEEC cells transfected with UCA1-expressing plasmids (UCA1-Exo) or negative control plasmids (Control- Exo). (**B**, **C**) Cell viability of EC18 and Kyse140 cells treated with exosomes derived from NEEC cells transfected with UCA1-expressing plasmids (UCA1-Exo) or negative control plasmids (Control- Exo). (**D**) Invasive ability of EC18 and Kyse140 cells treated with exosomes derived from NEEC cells transfected with UCA1-expressing plasmids (UCA1-Exo) or negative control plasmids (Control- Exo). Scale bar = 50 nm. (**E**) Migratory ability of EC18 and Kyse140 cells treated with exosomes derived from NEEC cells transfected with UCA1-expressing plasmids (UCA1-Exo) or negative control plasmids (Control- Exo). Scale bar = 50 nm. (**F**) Colony formation ability of EC18 and Kyse140 cells treated with exosomes derived from NEEC cells transfected with UCA1-expressing plasmids (UCA1-Exo) or negative control plasmids (Control- Exo). (*) denotes the difference between groups (*P*<0.05). Each experiment had a minimum of three replicates per treatment group.

### Effect of exosomal UCA1 on tumor growth *in vivo*

To investigate the effect of exosomal UCA1 *in vivo*, EC18 cells were transfected with UCA1-expressing vector (UCA1-vector) or negative control vector (Control), or UCA1-Exo and Control- Exo. Then, EC18 cells were injected subcutaneously into the right flank of male nude mice, and the tumor volumes were monitored every other day. In agree with findings *in vitro* experiments, the overexpression of UCA1 and UCA1-Exo significantly suppressed tumor growth, relative to tumors of mice treated with control or control-Exo (Figure 6A–6D), of which overexpression of UCA1 displayed more potent inhibitory effect than those of UCA1-Exo. Furthermore, H&E staining and immunohistochemistry assays were performed in mice tumor tissues, and the level of Ki67, a proliferation marker [28], was dramatically decreased in tumor tissues of mice treated with UCA1-vector and UCA1-Exo (Figure 6E, 6F). Growing evidence suggests that lncRNAs act as a competing endogenous RNA (ceRNA) to modulate the expression profile of targeting miRNAs [29]. To further determine the targeting miRNAs of UCA1, we carried out bioinformatics analysis and luciferase reporter assay (Figure 6G, 6H). The results showed that UCA1 directly targeted to miRNA-613, indicating that miRNA-613 might participate in the effect of UCA1 on esophageal cancer. Meanwhile, the level of miRNA-613 was higher in esophageal cancer tissues (Figure 6I), and the Pearson’s correlation analysis revealed that the negative correlation existed between miRNA-613 and UCA1 (Figure 6J).

**Figure 6:** **Effect of exosomal UCA1 on tumor growth *in vivo*.** (**A**) Representative images of nude mice treated with EC18 cells transfected with UCA1-expressing vector (UCA1-vector) or negative control vector (Control), or exosomes derived from NEEC cells transfected with UCA1-expressing plasmids (UCA1-Exo) or negative control plasmids (Control- Exo). (**B**) Tumor volumes of mice treated with EC18 cells transfected with UCA1-expressing vector (UCA1-vector) or negative control vector (Control), or exosomes derived from NEEC cells transfected with UCA1-expressing plasmids (UCA1-Exo) or negative control plasmids (Control- Exo). (**C**, **D**) Representative images of tumor tissues and tumor weights of mice treated with EC18 cells transfected with UCA1-expressing vector (UCA1-vector) or negative control vector (Control), or exosomes derived from NEEC cells transfected with UCA1-expressing plasmids (UCA1-Exo) or negative control plasmids (Control- Exo). (**E**) H&E staining assay for Ki67 expression in tumor tissues. (**F**) Immunohistochemistry assay for Ki67 expression in tumor tissues. (**G**) Putative binding site of miRNA-613 in UCA1. (**H**) Luciferase reporter assay. (**I**) Expression of miRNA-613 in esophageal cancer tissues (Tumor) and paired normal tissues (Control). (**J**) Pearson’s correlation between expressions of miRNA-613 and UCA1 in esophageal cancer tissues. (*) denotes the difference between groups (*P*<0.05). Each experiment had a minimum of three replicates per treatment group.

## DISCUSSION

Esophageal cancer, adenocarcinoma, and esophageal squamous cell carcinoma (ESCC) have emerged as the sixth leading cause of tumor-related death, and the eighth wide-spreading tumors all over the world [30]. Typically, esophageal cancer is diagnosed at an advanced phase due to the absence of evident early symptoms [31]. Thus, studying the mechanisms underlying the pathogenesis of esophageal cancer and exploring novel strategies for diagnosis and therapy are an urgent need. In the present study, we demonstrated that UCA1 was enriched in the exosomes from patients with esophageal cancer, and UCA1 was significantly decreased in both esophageal cancer tissues and the plasma. Also, exosomal UCA1 derived from NEECs could be internalized by esophageal cancer cells, thereby suppressing the malignant progression of recipient cancer cells through sponging miRNA-613. Furthermore, the anticancer effect of exosomal UCA1 inhibited tumor growth in vivo.

To date, multiple lncRNAs have been discovered to play an essential role in the development and progression of esophageal cancer [12, 32–34]. Given these observations, we selected twenty lncRNAs with critical regulatory functions in esophageal cancer and determined their expressions in tumor tissues. The results revealed that H19, MEG3, UCA1, and GAS5 were aberrantly expressed in esophageal cancer tissues, relative to adjacent normal tissues. Among these dysregulated lncRNAs, only UCA1 was significantly downregulated, which is consistent with the finding reported by Wang et al. [22]. Increasing evidence suggests that exosomal lncRNAs are representative of the physiological status of exosome-releasing cells, then impacting the cellular processes of recipient cells [35, 36]. In addition, exosomal lncRNAs have been reported as a potential biomarker for several cancers, such as colorectal cancer [37], gastric cancer [38], and prostate cancer [39]. Given such significant findings, we then attempted to determine the expression of UCA1 in plasma exosomes of patients with esophageal cancer. As observed in esophageal cancer tissues, we found that the expression of UCA1 was also decreased in plasma exosomes. Also, the downregulation of exosomal UCA1 was correlated with higher tumor and clinical grade.

Given the notable expression profile of UCA1 in esophageal cancer, we next carried out a series of assays to investigate the function of UCA1 in human esophageal cancer cells. As shown in our results, overexpression of UCA1 plays a significant inhibitory role in cell proliferation, migration, invasion, as well as colony formation, suggesting the anticancer role of UCA1 in esophageal cancer. A similar function of UCA1 is reported in esophageal squamous cell carcinoma (ESCC) [22]. In addition, UCA1 has been demonstrated to be essential for the effect of several antitumor medicines, such as metformin [40] and isorhapontigenin [41] in bladder cancer. On the other hand, there are more studies reporting the oncogenic role of UCA1 in several cancer types. For example, Tuo et al. reported that the upregulation of UCA1 promotes breast cancer cell growth and apoptosis through interacting with miRNA-143 [42]. Nie et al. also demonstrated that the overexpression of UCA1 is associated with increased cancer cell proliferation and colony formation in non-small cell lung cancer (NSCLC) [43]. Collectively, it is suggested that the role of UCA1, oncogenic or antitumor, displays cancer type-dependent patterns, which should be taken into account in the practical application.

Tumor tissue is a complex organ that is not only modulated by physiological activities of cancer cells themselves, but also by local extracellular, stromal cells, and distinct tissue architecture [44, 45]. Cell-to-cell communications within the cancer microenvironment play a critical role in the cell development and progression of cancer [46]. Of which, exosomes have been demonstrated to be essential extracellular messengers mediating intercellular interaction through transporting a cargo of bioactive components to neighboring cells, then influencing the recipient cells’ biochemical characteristics, signaling networks, and gene expression [44]. Over the past decade, numerous studies focus on the function of exosomal lncRNAs derived from tumor cells [47, 48], while a few attention has been drawn on exosomal lncRNAs released from the cancer microenvironment, such as normal cells. In this study, UCA1 was overexpressed in both NEEC and NEEC-Exo through transfecting with UCA1 vectors. Then, we found that NEEC-Exo could be internalized by in esophageal cancer cells and exerted antitumor role through inhibiting proliferation, migration, invasion, and colony formation of esophageal cancer cells. Furthermore, exosomal UCA1 suppressed tumor growth *in vivo*. Together, these results indicate that UCA1 can be shuttled from NEEC to esophageal cancer cells through exosome-mediated intercellular communication and plays an antitumor role in esophageal cancer in both *in vitro* and *in vivo*.

As an essential mechanism, lncRNAs act as a competing endogenous RNA (ceRNA), regulating the expression profile of targeting miRNAs [29]. To determine the mechanism underlying the effect of exosomal UCA1 in esophageal cancer, we identified that exosomal UCA1 competitively targeted to miRNA-613, through bioinformatics analysis and luciferase reporter assay. In papillary thyroid cancer, miRNA-613 is downregulated in cancer cells and inhibits cell growth, migration, and invasion through targeting sphingosine kinase 2 (SphK2) [49]. Also, miRNA-613 is associated with cell invasion and migration in triple-negative breast cancer through Daam1/RhoA signaling pathway [50]. To the best of our knowledge, the function of miRNA-613, to date, has not been intensively investigated in esophageal cancer. Thus, the observation in this study suggests that miRNA-613 may be a potential biomarker for esophageal cancer if the further comprehensive investigation is carried out.

## CONCLUSIONS

In conclusion, the results suggest that exosomal UCA1 derived from normal cells can be taken up by esophageal cancer cells, then attenuating tumor tumorigenesis and development *in vitro* and *in vivo*. Also, our observations demonstrated that exosomal UCA1 has a high diagnostic value for patients with esophageal cancer. Our study provides a new understanding of the carcinogenesis of esophageal cancer.

## MATERIALS AND METHODS

### Patients

The written informed consent was obtained from all subjects included in this study, and the study protocols were approved by the Ethics Committee of Gansu Provincial Hospital. The plasma samples were obtained from thirty patients with esophageal cancer and thirty healthy control subjects (Table 1). Fifteen paired esophageal cancer tissues and adjacent normal tissues were obtained from patients with esophageal cancer from the Gansu Provincial Hospital (Table 2).

**Table 2:** Clinical characteristics of paired esophageal cancer tissue samples.

**ID.**	**Age (years)**	**Sex**	**Smoking status**	**Tumor grade**	**Tumor stage**
1	76	Male	No	High grade	Non-muscle invasive
2	64	Female	Yes	Low grade	Invasive
3	61	Male	No	High grade	Non-muscle invasive
4	74	Female	No	Low grade	Invasive
5	64	Male	No	High grade	Non-muscle invasive
6	46	Female	No	Low grade	Non-muscle invasive
7	57	Male	Yes	High grade	Invasive
8	51	Female	Yes	Low grade	Non-muscle invasive
9	60	Male	No	High grade	Invasive
10	78	Female	Yes	High grade	Non-muscle invasive
11	75	Male	Yes	Low grade	Invasive
12	64	Male	Yes	High grade	Non-muscle invasive
13	51	Male	No	Low grade	Invasive
14	63	Female	No	High grade	Non-muscle invasive
15	77	Male	No	High grade	Non-muscle invasive

### Cell culture

Two esophageal cancer cell lines EC18 and Kyse140 and a normal esophageal cell line (NEEC) were purchased from Cell Bank of Type Culture Collection of the Chinese Academy of Sciences (Shanghai, China). Cells were cultured in RPMI-1640 medium (Thermo Fisher Scientific) supplemented with 10% fetal bovine serum (FBS) and 100 U/ml penicillin (Thermo Fisher Scientific) at 37° C with 5% CO_2_.

### Exosome isolation

Exosomes were isolated from the plasma and cell-cultured medium by ultracentrifugation-based assay [51, 52]. Briefly, the plasma and medium were centrifuged at 3000 g for 15 min to eliminate cells and cellular debris. Next, the supernatant was filtered through PVDF filter with 0.22 μm pore size (MilliporeSigma™). After the addition of Thrombin, the filtered plasma was centrifuged at 10,000 rpm for 5 min. Then, Thrombin-treated plasma and filtered culture medium were processed by ExoQuick exosome precipitation (System Biosciences) according to the manufacturer’s instruction.

### Transmission electron microscopy (TEM) and Nanoparticle tracking analysis (NTA)

Exosomes were fixed with 5% glutaraldehyde at incubation temperature and then maintained at 4° C. Then, exosomes were placed on the electron microscopy grids coated with Formvar cartion (Electron Microscopy Sciences) and incubated in 2% phosphotungstic acid solution for 30 s. Exosomes were imaged using a transmission electron microscope (Peabody, JEOL 100XCII). In addition, nanoparticle tracking analysis was carried out to determine the diameter and number of exosomes by using a NanoSight NS500 Instrument (NanoSight) according to the manufacturer’s instructions and previously described [53, 54].

### qRT-PCR

Total RNA was extracted from tissues, cells, and exosomes by using RNeasy Mini kit (Qiagen) according to the manufacturer’s instructions. cDNAs were synthesized by using High Capacity cDNA Reverse Transcription kit (Applied Biosystems) according to the manufacturer’s instructions. Quantitative real-time PCR reactions were performed by using SYBR Green assays (TaKaRa Biotechnology) on ABI 7900 system (Applied Biosystems). Primer sequence information was summarized in Table 3. GAPDH was used as a constitutive control, and relative expressions were analyzed using the 2^−ΔΔCt^ method [55].

**Table 3:** Primer information.

**Gene**	**Sequence (5’-3’)**	
**ANRIL**	**Forward**	TGCTCTATCCGCCAATCAGG
	Reverse	GGGCCTCAGTGGCACATACC
**CASC9**	Forward	TTGGTCAGCCACATTCATGGT
	Reverse	AGTGCCAATGACTCTCCAGC
**CCAT2**	Forward	CCACATCGCTCAGACACCAT
	Reverse	ACCAGGCGCCCAATACG
**FER1L4**	Forward	CCGTGTTGAGGTGCTGTTC
	Reverse	GGCAAGTCCACTGTCAGATG
**GAS5**	Forward	CACUCUGAGUGGGACAAGCUCUUCA
	Reverse	UGAAGAGCUUGUCCCACUCAGAGUG
**H19**	Forward	GCACCTTGGACATCTGGAGT
	Reverse	TTCTTTCCAGCCCTAGCTCA
**HNF1A-AS1**	Forward	AATCTCCTGCTGTCCTCTTC
	Reverse	AGGGCTCATCCTAACACTTT
**HOTAIR**	Forward	GGTAGAAAAAGCAACCACGAAGC
	Reverse	ACATAAACCTCTGTCTGTGAGTGCC
**MALAT1**	Forward	GTGAGCAAACTGTGTTGGCGTG
	Reverse	CATCGAGGTGAGGGGTGAAGGG
**MEG3**	Forward	GGGCATTAAGCCCTGACCTT
	Reverse	CCTTGGGGAGGGAAACACTC
**KCNQ1OT1**	Forward	CCAGCATAGCCTTATGGA
	Reverse	GCTGTCCGGGCCTCTGATCTCCGAT
**PCAT-1**	Forward	AATGGCATGAACCTGGGAGGCG
	Reverse	GGCTTTGGGAAGTGCTTTGGAG
**PEG10**	Forward	CATCCTTCCTGTCTTCGC
	Reverse	CCCTCTTCCACTCCTTCTTT
**SNHG1**	Forward	AGGCTGAAGTTACAGGTC
	Reverse	TTGGCTCCCAGTGTCTTA
**SNHG16**	Forward	ACAGGATGCCGTCTTGTGTT
	Reverse	GGTGGCAACCCATTAGCAGA
**SPRY4-IT1**	Forward	AGCCACATAAATTCAGCAGA
	Reverse	CGATGTAGTAGGATTCCTT TCA
**TP73-AS1**	Forward	CCGGTTTTCCAGTTCTTGCAC
	Reverse	GCCTCACAGGGAAACTTCATGC
**TUG1**	Forward	CTGAAGAAAGGCAACATC
	Reverse	GTAGGCTACTACAGGATTTG
**UBC1**	Forward	CCTGCTTGGAAACTAATGACC
	Reverse	AGGCTCAACTTCCCAGACTCA
**UCA1**	Forward	TTAAGGTGTCCACGCAGTCC
	Reverse	TGGGGATTACTGGGGTAGGG
**GAPDH**	Forward	CCGGGAAACTGTGGCGTGATGG
	Reverse	AGGTGGAGGAGTGGGTGTCGCTGTT
**MiRNA-613**	Forward	GTGAGTGCGTTTCCAAGTGT
	Reverse	TGAGTGGCAAAGAAGGAACAT
**U6**	Forward	CTCGCTTCGGCAGCACA
	Reverse	AACGCTTCACGAATTTGCGT

### Stability of exosomal UCA1

The plasma samples were placed at room temperature for 0 h, 8 h, 16 h, and 24 h, or were subjected to freezing-thawing cycles for 1, 2, 3, and 4 times between -20° C and room temperature. Then, exosomal RNAs were isolated from each plasma sample, and qRT-PCR analysis was carried out to measure the level of exosomal UCA1, following the method mentioned above.

### Western blots assay

Total proteins were extracted from exosomes by using cell lysis buffer (Beyotime Institute of Biotechnology), and the protein concentrations were measured by using the bicinchoninic acid (BCA) assay kit (SigmaAldrich). Total proteins were then separated by 12% polyacrylamide gel electrophoresis (SDS-PAGE) and were transferred to polyvinylidene difluoride (PVDF) membranes. Next, monoclonal rabbit anti-TSG101 and anti-CD63 (Santa Cruz) were used to incubated with membranes at 4° C overnight. After incubating with secondary antibodies for 1 hour at room temperature, membranes were visualized by enhanced chemiluminescence assays (Thermo Fisher Scientific). The optical densities of bands were analyzed using ImageJ software [56].

### Cell transfection

UCA1-expressing plasmid, negative control vector, and miRNA-613 mimics were synthesized by RiBoBio (Guangzhou, China). UCA1-expressing lentiviral vectors and negative control vector were synthesized by RiBoBio (Guangzhou, China). Cell transfection procedure was carried out using Lipofectamine 3000 (Invitrogen) according to the manufacturer’s instructions.

### Immunofluorescence

Exosomes (1 μg/ml) were suspended in 100 μl PBS solution with 1 ml PKH67 (Sigma). After incubation at room temperature for 4 min, bovine serum albumin (BSA) was added to terminate the staining process. Then, labeled exosomes were isolated using Exoquick exosome precipitation (System Biosciences), as mentioned above. Next, labeled exosomes were incubated with EC18, and Kyse140 cells labeled with DAPI (Thermo Fisher Scientific) at 37° C for 3 h. Immunofluorescence was imaged using a fluorescence microscope (Zeiss).

### Colony formation assay

EC18, and Kyse140 cells (1.0×10^5^) were transfected with UCA1-expressing plasmid or negative control vector or incubated with exosomes derived from NEEC cells transfected with UCA1-expressing plasmids or negative control plasmids. Then, cells were seeded in 6-well plates and cultured in RPMI-1640 medium (Thermo Fisher Scientific) supplemented with 10% fetal bovine serum (FBS) and 100 U/ml penicillin (Thermo Fisher Scientific) at 37° C with 5% CO_2_. After two weeks, the cell colonies were fixed using 95% methanol and stained using 0.1% crystal violet. The medium was replaced every three days.

### Cell invasion and migration assay

EC18, and Kyse140 cells (1.0× 10^5^) were transfected with UCA1-expressing plasmid or negative control vector or incubated with exosomes derived from NEEC cells transfected with UCA1-expressing plasmids or negative control plasmids. Cell invasion and migration assays were carried out as previously described [57, 58]. Cells were counted at five areas at random for each membrane.

### Cell proliferation assay

EC18, and Kyse140 cells (1.0× 10^5^) were transfected with UCA1-expressing plasmid or negative control vector or incubated with exosomes derived from NEEC cells transfected with UCA1-expressing plasmids or negative control plasmids. Cell proliferation assay was carried out by using Cell Counting Kit-8 (Abcam) according to the manufacturer’s instruction. The absorbance was measured at 450 nm by using a spectrophotometer (Tecan).

### Animal models

All animal experiments were approved by the Institutional Animal Care and Use Committee of Gansu Provincial Hospital. EC18 cells (1 × 10^6^) were transfected with UCA1-expressing vector (UCA1-vector) or negative control vector (Control) and then injected subcutaneously into the right flank of male nude C57BL/6 mice (6 week-old; 34.6 ± 1.2 g; n=6). Tumor volumes were monitored every other day. Two weeks post-injection, mice were sacrificed, and tumor size and weight were recorded. In another experiment, EC18 cells (1 × 10^6^) were injected subcutaneously into the right flank of male nude C57BL/6 mice (6 week-old; 35.1 ± 1.8 g; n=6). When tumor volumes reached around 0.1 cm^3^, exosomes derived from NEEC cells transfected with UCA1-expressing plasmids (UCA1-Exo) or negative control plasmids (Control- Exo) were injected directly into tumors every other day. After 15 days, mice were sacrificed, and tumor size and weight were recorded.

### Immunohistochemistry

Hematoxylin and eosin (H&E) staining and IHC staining were carried out to detect the expression of Ki67, as previously described [59, 60]. Anti-Ki67 antibody (Abcam) was used to immunohistochemistry assay.

### Luciferase reporter assay

The plasmids carrying the putative binding site of miRNA-613 were synthesized from the 3’UTR of UCA1 and then inserted into the firefly luciferase reporter gene in pMIR (Ambion). The plasmids carrying mutated miRNA-613 binding site were inserted into the same luciferase reporter to test binding specificity. Next, the plasmids were transfected with miRNA-613 mimic or miRNA negative control (miRNA-NC) into EC18 cells by using the Lipofectamine™ 3000 kit (Invitrogen) according to the manufacturer’s instructions. After 24 h, relative luciferase levels were measured using the luciferase assay kit (Promega).

### Statistical analysis

Data were represented as mean ± S.D and analyzed by SPSS 19.0 software (SPSS Inc, Chicago, USA). Mean differences between groups were analyzed using the Tukey’s test. The differences in characteristics between healthy controls and esophageal cancer cases were determined by using Pearson’s χ2 test. The receiver operating characteristic (ROC) curve was analyzed using Graphpad software (version 6.0) [61]. Statistical differences were defined as P < 0.05.
